RETRACTED

# IL-21 Regulates the Differentiation of a Human γδ T Cell Subset Equipped with B Cell Helper Activity

**DOI:** 10.1371/journal.pone.0041940

**Published:** 2012-07-25

**Authors:** Nadia Caccamo, Matilde Todaro, Marco P. La Manna, Guido Sireci, Giorgio Stassi, Francesco Dieli

**Affiliations:** 1 Dipartimento di Biopatologia e Biotecnologie Mediche e Forensi, Università degli Studi di Palermo, Palermo, Italy; 2 Dipartimento di Discipline Chirurgiche ed Oncologiche, Università degli Studi di Palermo, Palermo, Italy; French National Centre for Scientific Research, France

## Abstract

Vγ9Vδ2 T lymphocytes recognize nonpeptidic antigens without presentation by MHC molecules and display pleiotropic features. Here we report that coculture of Vγ9Vδ2 cells with phosphoantigen and IL-21 leads to selective expression of the transcription repressor Bcl-6 and polarization toward a lymphocyte subset displaying features of follicular B-helper T (T_FH_) cells. T_FH_-like Vγ9Vδ2 cells have a predominant central memory (CD27^+^CD45RA^−^) phenotype and express ICOS, CD40L and CXCR5. Upon antigen activation, they secrete IL-4, IL-10 and CXCL13, and provide B-cell help for antibody production *in vitro*. Our findings delineate a subset of human Vγ9Vδ2 lymphocytes, which, upon interaction with IL-21-producing CD4 T_FH_ cells and B cells in secondary lymphoid organs, is implicated in the production of high affinity antibodies against microbial pathogens.

## Introduction

Development of efficient humoral immune response results in the production of a high-affinity antibodies that are essential for the clearance of many infectious pathogens. Generation of these protective antibodies takes place in specialized structures in secondary lymphoid organs, known as germinal centers (GCs), and requires the combination of diverse events such as isotype-switch, somatic hypermutation and affinity maturation, which occur upon interaction between activated B lymphocytes and CD4 follicular helper T (T_FH_) lymphocytes [1], [2]. T_FH_ cells are defined by follicular localization and high expression of specific markers [3]–[7]: CXCR5 that drives T_FH_ cells to migrate into the B cell follicles; the inhibitory receptor PD-1 and the costimulatory molecule ICOS, which interact with their corresponding ligands on B lymphocytes; the signature cytokine IL-21, which predominantly acts as a paracrine factor for GC B lymphocytes, but has only limited autocrine function as regulator of T_FH_ lineage fate. The transcriptional repressor Bcl-6 is a crucial intrinsic regulator of T_FH_ lineage commitment, but the differentiation pathway from naive CD4 to T_FH_ cells is the subject of intense studies.

RETRACTED

Despite CD4 T_FH_ cells, other T cell subsets including CD8 T cells, NKT cells and γδ T cells are capable to provide B cell help and as such contribute to the outcome of antibody response [8]–[10]. Early studies in αβ T cell–deficient mice demonstrated a nonredundant role for γδ T cells in the generation of antimicrobial antibodies [11], [12] and autoantibodies [13]–[15]. However, the finding that γδ T cell-deficient mice do not show marked defects in IgM and IgG production, suggested that γδ T cells may have a modulatory, rather then a primary function in the control of humoral immunity. Antibody production was also increased in *in vitro* cultures of human γδ T cells with B cells [16], [17], but the amount of secreted antibody was low and the mechanisms underlying the observed B-cell help were not examined. More recent studies have shown that human γδ T cells are found in secondary lymphoid tissues [18], [19], where they are scattered throughout the T zone and clustered within follicles [20], express costimulatory molecules after TCR-triggering and provide B-cell help *in vitro*, suggesting their participation in humoral immunity [20].

The majority of human peripheral blood γδ T cells, express a TCR consisting of the Vγ9 and the Vδ2 chains (here and thereafter referred to as Vγ9Vδ2 cells) and recognize nonpeptidic phosphorylated metabolites of isoprenoid biosynthesis produced by microorganisms and stressed cells [21]–[23]. Upon activation, Vγ9Vδ2 cells can be skewed toward distinct effector functions depending on polarizing cytokines, in analogy to CD4 helper T cells [24]–[26]. Accordingly, under appropriate culture conditions, Vγ9Vδ2 cells divert from the typical Th1-like phenotype and polarize to Th2 [26], [27], Th17 [28], [29] and Treg cells [30]. Such a broad plasticity emphasizes the capacity of Vγ9Vδ2 cells to influence the nature of immune response to different challenges.

We and others have shown that antigen-stimulated Vγ9Vδ2 cells acquire T_FH_-associated features (ICOS, CD40L and CXCR5 surface expression, *IL-21R* mRNA expression, IL-4 and IL-10 secretion) and provide B-cell help for antibody production [30], [25], [31]; moreover, a recent study by Bansal *et al.* [32], reported that Vγ9Vδ2 T cells stimulated with the phosphoantigen HMB-PP in the presence of IL-21, express markers associated with T_FH_ cells and support antibody production by B cells, clearly pointing to IL-21 as the key cytokine for differentiation of this T_FH_-like Vγ9Vδ2 cell subset.

Yet no data are available on the relative role of antigen and cytokines for the regulation of lineage-specifying factors required for the differentiation of T_FH_ Vγ9Vδ2 cells.

We show here that in human Vγ9Vδ2 cells, Bcl-6 expression and polarization towards T_FH_ cells are efficiently induced by coordinated TCR triggering and IL-21. Moreover, we provide detailed phenotypic and functional analysis of T_FH_-like Vγ9Vδ2 cells, and in agreement with the study of Bansal et al. [32], suggest that the interaction between Vγ9Vδ2 T_FH_ cells, CD4 T_FH_ cells and B cells in reactive secondary lymphoid tissues may profoundly impact on the production of high affinity antibodies against microbial pathogens.

RETRACTED

## Methods

### Subjects

Peripheral blood mononuclear cells (PBMC) were isolated from buffy coats of healthy volounteers by density gradient centrifugation using Ficoll-Hypaque (Pharmacia Biotech, Uppsala, Sweden). PBMC and mononuclear cells were also isolated from fresh tonsils of patients undergoing tonsillectomy. According to Italian rules (art. 13, DLgs n. 196/03), this study did not require authorisation by the local ethical committee. The study was performed in accordance to the principles of the Helsinki declaration and all individuals gave written informed consent to participate.

### Cell Purification and Culture

Peripheral blood CD14^+^ monocytes and Vγ9Vδ2 cells were isolated by positive selection with CD14- and Vδ2-specific microbeads, respectively (Miltenyi Biotec, Bergisch Gladbach, Germany). Dendritic cells (DCs) were obtained from sorted CD14^+^ monocytes after culture for 5–6 days in the presence of 25 ng/ml GM-CSF and 1000 U/ml IL-4 (both from Euroclone, Milan, Italy). Subsets of Vγ9Vδ2 cells were isolated to over 99% purity of total Vγ9Vδ2 T cells, after staining with phycoerythrin (PE)-conjugated anti-CD27 (1A4, BD Biosciences, San Josè, CA) and allophycocyanin (APC)-conjugated anti-CD45RA (M-T271, BD Biosciences) monoclonal antibodies (mAbs), followed by cell sorting with a FACSAria (BD Biosciences). Sorted Vγ9Vδ2 T cell subsets were labeled with CFSE (Molecular Probes, Eugene, OR) and were cultured in RPMI-1640 medium (Euroclone, Milan, Italy) supplemented with 2 mM L-glutamine, 20 nM Hepes buffer, 10 µg/ml gentamycin, 100 U/ml penicillin/streptomycin (Sigma-Aldrich, St. Louis, MO) and 10% pooled human AB^+^ serum (kindly provided by the Blood Bank of the University Hospital, Palermo), and 5×10^4^ cells were cultured in U-bottom 96-well plates, with an equal number of irradiated (30 Gy from a cesium source) DCs and isopentenyl pyrophosphate (IPP; Sigma-Aldrich; 10^−5^ M final concentration). After 48 hrs, recombinant human cytokines were added to cultures: IL-2 (Novartis Pharma; 50 IU/ml final concentration), or recombinant IL-15 (10 ng final concentration, R&D Systems), or recombinant IL-21 (100 ng/ml final concentration, eBioscience through Prodotti Gianni, Mlan, Italy). Every three days, half of the medium was removed and replaced with fresh medium containing the recombinant cytokine. The cells were harvested, following 9–12 days of culture.

RETRACTED

### FACS Staining and Sorting

The following conjugated antibodies were used in different combinations: anti-Vδ2 (B6, BD Biosciences), anti-Vγ9 (B3, BD Biosciences), anti-CD27 (1A4, BD Biosciences), anti-CD45RA (M-T271, BD Biosciences), anti-CD25 (M-A251, BD Pharmingen), anti-CCR7 (a gift of Dr. M. Lipp, Max-Delbruch-Center for Molecular Medicine, Berlin, Germany), anti-HLA-DR monomorphic (a gift of Prof. V. Horejsi, Institute of Molecular Genetics, Academy of Science of the Czech Republic, Prague), anti-ICOS (a generous gift of Dr. R.A. Kroczek), anti-CD40L (TRAP1, BD Biosciences), anti-CCR3 (61828.111, R&D Systems), anti-CCR4 (1G1, BD Biosciences), anti-CCR5 (2D7, BD Bioscences), anti-CCR6 (11A9, BD Biosciences), anti-CXCR3 (1C6/CXCR3, BD Biosciences), anti-CXCR5 (a gift of Dr. R. Keoczek, Molecular Immunology, Robert Koch Institute, Berlin, Germany) and isotype control mAbs. Vγ9Vδ2 cells were incubated in U-bottom 96-well plates with labelled mAbs in PBS containing 1% FCS, for 30 min at 4°C according to manufacturers’ recommendations, washed, and analyzed by flow cytometry on an FACSCalibur or FACSCanto II (BD Biosciences) and analyzed with FlowJo software (Tree Star). Viable cells were gated by forward and side scatter, and the analysis was performed on 100,000 acquired events for each sample.

### Proliferation, Cytokine Analysis and Chemotaxis Assay

Proliferation of primed Vγ9Vδ2 cells was assessed 72 hours after stimulation of cells (10^5^/ml) with IPP (10^−5^ M final concentration) and irradiated DCs and measured by CFSE dilution. The cytokine-producing capacity of primed Vγ9Vδ2 cells was assessed by stimulation of cells (10^5^/ml) for 24 hrs with IPP (10^−5^ M final concentration) and irradiated DCs. Cytokines (TNF-α, IFN-γ, IL-2, IL-4, IL-10 and IL-17) and chemokine (CXCL13) in culture supernatants were measured by ELISA, according to the manufacturer’s instructions (R&D Systems). Intracellular staining for IFN-γ, IL-4, IL-10 and IL-17 was done on Vγ9Vδ2 cells stimulated for 6 hrs with IPP (10^−5^ M final concentration) in the presence of GolgiStop (BD Biosciences) for the final 4 hrs of culture. Cells were fixed and made permeable with BD Cytofix/Cytoperm Plus (BD Biosciences) according to the manufacturer’s instructions. Cells were incubated with fluorescein isothiocyanate (FITC)-labeled anti-IFN-γ mAb (B27, BD Biosciences), PE-labelled anti-IL-4 mAb (8D4-8, BD Biosciences), PE labeled anti-IL-10 mAb (JES5-16E3, BD Biosciences) and APC-labeled anti-IL-17 mAb (eBIO64-DEC17, eBioscience), or isotype-control mAbs. Cells were washed and data were acquired on a FACSCalibur or FACSCanto II (BD Biosciences) and analyzed with FlowJo software (Tree Star).

RETRACTED

The chemotactic ability of IL-21-primed Vγ9Vδ2 cells was assayed using a double-chamber system with 3-µm pores (Transwell, Costar), according to [31]. Briefly, 10^5^ Vγ9Vδ2 cells were added to the upper chamber and recombinant human CXCL13 (R&D Systems, 3 µM final concentration) to the lower chamber and incubated at 37°C for 2 h in a 5% CO_2_ humidified incubator. In some experiments, anti-CXCR5 or isotype control mAbs were added to the lower chamber during the test. Assays were performed in triplicate. Afterward, the membrane was removed, washed on the upper side with PBS, fixed, and stained. Migrated cells were counted microscopically at x1000 magnification in five randomly selected fields per well. Percentage migration was calculated by measuring the counts recovered from the lower chamber and comparing them to the total input counts. Results represent the mean ± SD of three independent experiments.

### Antibody Production *in vitro*

Vγ9Vδ2 T cell help in antibody production was studied as follows. IL-21-primed Vγ9Vδ2 T cells were co-cultured with sorted tonsillar B cells in 96-well plates at 10^5^ cells/well each of T and B cells in the presence or absence of IPP, in RPMI 1640 medium supplemented with 10% heat-inactivated FCS (Euroclone), 2 mM L-glutamine, 20 nM HEPES and 100 U/ml penicillin/streptomycin. 10 days later IgM, IgG, and IgA levels in the culture supernatants were determined by ELISA.

### Real-time Quantitative RT-PCR

Total RNA was extracted with the ABI PRISM 6100 Nucleic Acid PrepStation (Perkin-Elmer Applied Biosystems) according to the manufacturer’s instructions. Random hexamers and an MMLV Reverse Transcriptase kit (Stratagene, La Jolla, CA) were used for cDNA synthesis. Transcripts were quantified by real-time quantitative PCR on an ABI PRISM 7700 Sequence Detector (Perkin-Elmer Applied Biosystems) with Applied Biosystems predesigned TaqMan Gene Expression Assays and reagents according to the manufacturer’ s instructions. The following probes were used (identified by Applied Biosystems assay identification number): *RORC*, Hs01076112_m1; *TBX21*, Hs00203436_m1; *BCL6*, Hs00277037_m1; *GATA3*, Hs00231122_m1; *IL21R*, Hs00222310_m1; *IFNG*, HS00174143_m1; *IL-4*, HS00174122_m1; *IL-10*, HS00174086_m1; *IL-13*, HS00174379_m1; *IL-21*, Hs00222327_m1. For each sample, mRNA abundance was normalized to the amount of 18S rRNA.

### Statistics

A standard two-tailed *t*-test or a *t*-test with Welch’s correction was used for statistical analysis. P values of <0.05 were considered significant.

RETRACTED

## Results

### Factors Inducing the Differentiation of Vγ9Vδ2 T_FH_ Cells

It has been previously shown that antigen-stimulated Vγ9Vδ2 cells acquire T_FH_-associated features (ICOS, CD40L and CXCR5 surface expression, IL-4 and IL-10 secretion and B-cell help for antibody production) [20], [25], [31], including expression of *IL-21R* mRNA [25], yet no data are available on the antigen and cytokine requirements for the differentiation of this subset of T_FH_ Vγ9Vδ2 cells. To identify conditions that permit the polarization of human T_FH_ Vγ9Vδ2 cells, we stimulated highly purified subsets of naive (T_naive_, CD45RA^+^CD27^+^), central memory (T_CM_, CD45RA^−^CD27^+^), effector memory (T_EM_, CD45RA^−^CD27^−^) and terminally-differentiated effector memory (T_EMRA_, CD45RA^+^CD27^−^) Vγ9Vδ2 cells with irradiated autologous DCs and antigen (IPP), together with different cytokines (see Materials and Methods for details), and analyzed their surface marker expression. Primarily, we used ICOS expression as a signature of T_FH_ Vγ9Vδ2 cells because (a) expression of high levels of ICOS is a defining feature of CD4 T_FH_ cells [33], (b) ICOS is not expressed by resting Vγ9Vδ2 cells and (c) the ability of CD4 [34] and Vγ9Vδ2 [31] T_FH_ cells to help B cells is mediated by ICOS.

In the absence of exogenous cytokines, only a small percentage (2% or less) of antigen-primed Vγ9Vδ2 cells expressed ICOS. Addition of IL-2 or IL-15 did not enhance ICOS expression (**Figure 1A**), but addition to cultures of IL-21 strongly induced expression of ICOS on the majority of Vγ9Vδ2 T cells (**Figure 1A**). Vγ9Vδ2 cells with a T_naive_ and a T_CM_ phenotype were the only subsets that can be polarized to ICOS expression upon culture with antigen and IL-21, while T_EM_ and T_EMRA_ Vγ9Vδ2 cells failed to express any of the tested T_FH_ surface markers under similar cytokine priming conditions (**Figure 1B**). Therefore, in subsequent *in vitro* culture experiments we used sorted CD27^+^ Vγ9Vδ2 T cells (which contains both T_naive_ and a T_CM_ cells) as a starting population.

**Figure 1:** Surface phenotype of Vγ9Vδ2 T cells differentiated by antigen and IL-21. Vγ9Vδ2 T cells were primed for 12 days with an equal number of irradiated DCs and IPP, in the presence of IL-21. Cells were surface stained for several different markers. (A) shows CD27 and ICOS expression on Vγ9Vδ2 T cells that had been cultured with antigen alone (Nil) or with antigen but in the presence of IL-2, IL-15 or IL-21. Data are representative of seven independent experiments, each carried out in triplicate. (B) FACS analysis to determine the percentage of ICOS^+^ Vγ9Vδ2 T cells among highly purified T_Naive_,T_CM_, T_EM_ and T_EMRA_ subsets Vγ9Vδ2 T cells from eight different donors, primed with antigen and IL-21. Each symbol represents a single donor, small horizontal bars indicate the mean. In (C), expression of activation and costimulatory molecules, and chemokine receptors is shown upon gating on Vγ9Vδ2 T cells. The vertical line in each panel indicates the negative cut-off as determined by staining with isotype-control mAbs. (D) Time-course of ICOS expression on Vγ9Vδ2 T cells that had been cultured with medium alone (filled squares), with IL-21 alone (filled circles) or with antigen but in the absence (open circles) or presence (open squares) of IL-21. Data are representative of five independent experiments each carried out in triplicate.

RETRACTED

The vast majority of Vγ9Vδ2 T cells differentiated in the presence of antigen and IL-21 had a predominant central memory phenotype as they did not express CD45RA, but expressed CD27. Moreover, they expressed the activation markers CD25 and HLA-DR, and the costimulatory molecules CD40L and ICOS. They also expressed low levels CXCR5, but they did not express CXCR3, CCR3, CCR5 and CCR6 (**Figure 1C**).

Time-course experiments showed, that ICOS expression by Vγ9Vδ2 T cells differentiated in the presence of antigen and IL-21 was evident after 2 days of culture, reached a peak at day 4–6 and declined by day 8 onwards (**Figure 1D**).

### The Relative Role of Antigen and IL-21 in the Regulation of Lineage-specifying Factors

Bcl-6 was recently identified as a master regulator of T_FH_ differentiation [35]–[37]. We therefore measured the expression of mRNA encoding human Bcl-6 (*BCL6*) in Vγ9Vδ2 T_FH_ cells. Culture of sorted Vγ9Vδ2 T cells with antigen and IL-21 induced high expression of *BCL6*, while expression of *RORC* (RORγt), *TBX21* (T-bet) and *GATA3* was induced only slightly or not at all (**Figure 2A**). Addition of IL-1β, IL-2, IL-6, IL-12, IL-15 or TGFβ, either alone, or in combination with IL-21 (data not shown), to cultures of Vγ9Vδ2 T cells and antigen did not induce *BCL6* expression (**Figure 2B**).

**Figure 2:** Antigen and IL-21 differently regulate expression of lineage-specifying transcription factors in Vγ9Vδ2 T cells. Vγ9Vδ2 T cells were cultured with an equal number of irradiated DCs and IPP, in the presence of IL-21. (A) RT-PCR of the expression of *RORC*, *TBX21, GATA3* and *BCL6* in cells primed with antigen in the absence (white columns) or presence (black columns) of IL-21. (B) RT-PCR of the expression of *BCL6* on Vγ9Vδ2 T cells that had been cultured with antigen in the presence of different cytokines. (C) and (D), RT-PCR of the expression of *IL21R* (C) and *BCL6* (D), in Vγ9Vδ2 T cells primed for various times (horizontal axes) with medium (filled circles), with IL-21 alone (open circles) or with antigen but in the absence (filled squares) or presence (open squares) of IL-21. Data represent the mean values ± SD of five separate experiments, each carried out with cells from three different donors.

RETRACTED

To investigate early events in the differentiation of Vγ9Vδ2 T_FH_ cells and the relative role of antigen and the polarizing cytokine IL-21, we assessed the kinetics of expression of mRNA encoding for *IL-21R* and *BCL6*. Data are shown in **Figure 2C and 2D**, respectively. Resting, unstimulated Vγ9Vδ2 T cells do not constitutively express both *IL21R* and *BCL6*. Vγ9Vδ2 TCR stimulation by antigen induced expression of *IL21R* mRNA, as early as 6 hrs after stimulation. Expression of *IL21R* mRNA peaked on day 2–3 and consistently decreased on day 6. Antigen stimulation alone was not sufficient to induce detectable *BCL6*, indicating that upregulation of lineage-specifying transcription factors requires combination of antigen and IL-21. Accordingly, *BCL6* was significantly induced by antigen in the presence of IL-21, which peaked on days 3–6 and decreased by day 9 onwards.

These results indicate that the coordinated combination of TCR triggering by antigen and the presence of IL-21, induces sustained expression of *BCL6* in human Vγ9Vδ2 T cells, which is consistent with their ability to promote differentiation and polarization towards T_FH_ cells.

### Proliferation Potential and Cytokine Production of Vγ9Vδ2 T_FH_ Cells

In the following set of experiments, we assessed the proliferation potential of purified Vγ9Vδ2 T_FH_. To this end, we generated *in vitro* Vγ9Vδ2 T_FH_ cells with antigen and IL-21, as previously described. Vγ9Vδ2 T_FH_ cells were sorted, labelled with CFSE and stimulated again *in vitro* with IPP in the presence of irradiated DCs. As shown in **Figure 3A**, proliferation of Vγ9Vδ2 T_FH_ cells was very low in the presence of DCs, but without antigen. As expected, upon stimulation with antigen and DCs, or with immobilized anti-CD3 mAb, Vγ9Vδ2 T_FH_ cells, showed significant proliferation, indicating that they have an high proliferative potential to TCR ligands, and suggesting that they are at an early stage of memory cell differentiation.

**Figure 3:** Proliferation and cytokine production of Vγ9Vδ2 T_FH_ cells. Vγ9Vδ2 T_FH_ cells were obtained upon culture with antigen and IL-21, as previously described. Vγ9Vδ2 T_FH_ cells were sorted, labelled with CFSE and re-stimulated *in vitro* with IPP in the presence of irradiated DCs. (A) Proliferation was measured by CFSE dilution, after 72 hrs stimulation. Cytokine levels were assessed by ELISA (B) or intracellular FACS analysis (C), 24 and 6 hrs after stimulation, respectively. Numbers in the quadrant of dot plots in Figure 3C indicate the percentages of positive cells. (D) RT-PCR of the expression of *IL4, IL10, IL13, IL17, IL21* and *IFNG* in Vγ9Vδ2 T_FH_ cells stimulated *in vitro* with IPP in the presence of irradiated DCs for 6 hrs. The Figure shows one out of five independent experiments.

RETRACTED

We then studied the pattern of cytokine production in Vγ9Vδ2 T_FH_ cells, after a 24 hrs stimulation period with antigen and DCs *in vitro*. As shown in **Figure 3B**, Vγ9Vδ2 T_FH_ cells produced very few, if any, amounts of cytokines upon stimulation with DCs, but in the absence of antigen. However, Vγ9Vδ2 T_FH_ cells that had been stimulated by antigen and DCs, produced IL-2, IL-4 and, to a lower extent, IL-10, but not IFN-γ, TNF-α or IL-17. Moreover, and differently than CD4 T_FH_ cells, Vγ9Vδ2 T cells cultured with antigen and IL-21 did not produce IL-21, in agreement with previously published results [25].

This pattern of cytokine production was confirmed by flow cytometry studies in Vγ9Vδ2 T_FH_ cells 6 hrs after *in vitro* culture with antigen and DCs: as expected from the ELISA data, antigen-stimulated Vγ9Vδ2 T cells expressed IL-4 and IL-10, but not IFN-γ or IL-17 (**Figure 3C**).

Given that Vγ9Vδ2 T_FH_ cells are capable of producing the Th2 cytokines, IL-4 and IL-10 in the spite of very low, if any, GATA-3 expression, we analysed whether this pattern involved other Th2 cytokines. In agreement with the ELISA and flow cytometry data, antigen-stimulated Vγ9Vδ2 T_FH_ cells expressed *IL-4* and *IL-10* mRNA, but not *IL-13* mRNA (**Figure 3D**). Moreover, and as expected, antigen-stimulated Vγ9Vδ2 T_FH_ cells did not express both *IL-13*, *IFNG* and *IL-21* mRNA.

Thus Vγ9Vδ2 T_FH_ cells are characterized by the distinctive pattern of IL-4 and IL-10 expression in the absence of significant GATA-3 and IL-13 expression. Finally, and differently than CD4 T_FH_ cells, Vγ9Vδ2 T_FH_ cells neither express nor produce IL-21.

### Chemokine Production and Migratory Properties of Vγ9Vδ2 T_FH_ Cells

It has been previously demonstrated that Vγ9Vδ2 T cells stimulated with HMB-PP in the presence of IL-21, but not of IL-2 or IL-4, express CXCL13 mRNA, and the secretion of CXCL13 by PBMC stimulated with antigen and IL-21 depends on the presence of Vγ9Vδ2 T cells [25]. Data reported in **Figure 4A** confirm that Vγ9Vδ2 T_FH_ cells stimulated by IPP and DCs, secrete CXCL13 into the supernatant.

**Figure 4:** Production of CXCL13 and migration to CXCL13 Vγ9Vδ2 T_FH_ cells. Vγ9Vδ2 T_FH_ cells were obtained upon culture with antigen and IL-21, as previously described. In (A), Vγ9Vδ2 T_FH_ cells were sorted and re-stimulated *in vitro* with IPP in the presence of irradiated DCs. Supernatants were collected after 24 hrs stimulation and CXCL13 levels assessed by ELISA. In (B) Vγ9Vδ2 T_FH_ cells were tested for *in vitro* migration to CXCL13 (3 µM, final concentration) in the absence or presence of anti-CXCR5 or isotype-matched control mAbs (15 µg/ml, final concentration). Data are representative of three independent experiments. *p<0.02 when compared with groups consisting of Vγ9Vδ2 T_FH_ cells migrating to CXCL13 in the absence of any Ab or in the presence of isotype-matched control mAb.

RETRACTED

The finding that IL-21-primed Vγ9Vδ2 T_FH_ cells express low levels of CXCR5 led us to explore if the expressed CXCR5 is functional, by assessing migration in response to the CXCR5 ligand, CXCL13 in a 2 hrs assay. IL-21-primed Vγ9Vδ2 T_FH_ cells migrated readily in response to CXCL13 (**Figure 4B**), but migration was significantly inhibited by an anti-CXCR5 mAb added to cultures (**Figure 4B**), indicating that the expressed CXCR5 receptor is functional.

### Vγ9Vδ2 T_FH_ Cells Help B Cells for Antibody Production

As Vγ9Vδ2 T_FH_ cells express costimulatory molecules and produce IL-4 and IL-10 upon antigen stimulation, we tested whether or not these cells were able to support B cells to secrete immunoglobulins. To this end, we generated *in vitro* Vγ9Vδ2 T_FH_ cells with IPP and IL-21, as previously described. Vγ9Vδ2 T_FH_ cells were sorted, and cultured with CD19 B cells isolated from the tonsil of the same donor, in the presence or absence of antigen. As shown in **Figure 5**, B cells produced comparable low amounts of IgA, IgG and IgM when cultured for 10 days without Vγ9Vδ2 T cells, but co-culture of B cells with Vγ9Vδ2 T_FH_ cells and IPP resulted in an 15-fold increase in the production of IgG, a 10-fold increase in the production of IgA and a 5-fold increase in the production of IgM. Of note, Vγ9Vδ2 T_FH_ cells failed to cause significant increase of antibody production in co-cultures with B cells carried out in the absence of antigen.

**Figure 5:** Vγ9Vδ2 T_FH_ cells help B cells for antibody production. Vγ9Vδ2 T cells were cultured with an equal number of irradiated DCs and IPP, in the presence of IL-21. At the end of culture, Vγ9Vδ2 T_FH_ cells were sorted, and cultured with CD19 B cells isolated from the tonsil of the same donor, in the presence or absence of IPP. Ten days later, total IgG, IgA and IgM levels in culture supernatants were assessed by ELISA. *p<0.001 and **p<0.02 when compared with the group consisting of B cells cultured with Vγ9Vδ2 T_FH_ cells but in the absence of antigen. One out of five independent experiments is shown.

RETRACTED

The B cell helper activity of Vγ9Vδ2 T_FH_ cells in *in vitro* co-cultures was strictly dependent on their provision of both costimulatory molecules and cytokines. In fact, blocking of CD40L or ICOS caused a drastic reduction of both IgG and IgA production (**Figure 6**). Similarly, addition to co-cultures of antibodies neutralizing IL-4 and IL-10 caused reduction of IgG production, while a modest, not significant decrease of IgA production was only observed upon neutralization of IL-10, but not of IL-4 (**Figure 6**).

**Figure 6:** Vγ9Vδ2 T_FH_ cell helper activity requires costimulatory molecules and cytokines. Vγ9Vδ2 T cells were cultured with an equal number of irradiated DCs and IPP, in the presence of IL-21. At the end of culture, Vγ9Vδ2 T_FH_ cells were sorted and cultured with CD19 B cells isolated from the tonsil of the same donor, in the presence of IPP and mAbs to costimulatory molecules or cytokines (see Materials and Methods). Ten days later, total IgG and IgA levels in culture supernatants were assessed by ELISA. *p<0.005 and **p<0.02 when compared with the group consisting of B cells cultured with Vγ9Vδ2 T_FH_ cells and antigen. One out of five independent experiments is shown.

These data therefore suggest that antigen stimulation in the presence of IL-21 induces a population of Vγ9Vδ2 T_FH_ cells which supplies B cells with costimulatory signals and cytokines required for immunoglobulin production.

## Discussion

Vγ9Vδ2 T cells display *in vitro* a certain degree of plasticity in their function, that is reminiscent of conventional CD4 T cells. In analogy with CD4 T cells, where a plethora of specialized subsets affect the host’s response, Vγ9Vδ2 T cells may readily and rapidly assume distinct Th1-, Th2-, Th17- and Treg-like effector functions, [24]–[30] suggesting that they profoundly influence cell-mediated immune responses. Comparatively, little is known about their role in antibody-mediated immune responses.

We [31] and others [20], [25] previously identified a unique subset of peripheral blood and tonsil Vγ9Vδ2 cells with T_FH_-like properties, which upon antigen stimulation express ICOS, CD40L, CXCR5, and IL-21R, secrete IL-4 and IL-10 and provide B-cell help for antibody production *in vitro*, but the cytokine requirements for differentiation of this T_FH_-like Vγ9Vδ2 cell subset have not been examined yet.

Here we show that in human Vγ9Vδ2 T cells, Bcl-6 expression and polarization towards a T_FH_-like phenotype is efficiently induced by coordinated antigen stimulation of the specific TCR and IL-21. The *in vitro* differentiated Vγ9Vδ2 T_FH_ cells exhibit a T_CM_ phenotype, illustrated by the expression of CD27 in the absence of CD45RA. Vγ9Vδ2 T_FH_ cells distinctively express both activation (CD25 and HLA-DR) and costimulatory (CD40L and ICOS) molecules and also express, although at low levels, CXCR5, a chemokine receptor that has been identified as a marker of T_FH_ cells [1], [2], but they do not express any other tested chemokine receptor (CXCR3, CCR3, CCR4, CCR5, and CCR6). Conversely, Th1-like Vγ9Vδ2 T cells express CXCR3 and CCR5 [19], and Th17-like Vγ9Vδ2 T cells express CCR6 [29]. Expression of CXCR5 on human Vγ9Vδ2 T_FH_ cells is a matter of debate. Brandes and colleagues [20] did not detect CXCR5 expression on both peripheral blood and tonsillar Vγ9Vδ2 T cells, while other studies [31], [38] found this receptor being expressed by a subset of Vγ9Vδ2 T_FH_. Moreover, Forster et al. [39] found that in healthy individuals, 2% of peripheral blood γδ T cells, but ∼23% of tonsillar γδ T cells express CXCR5 and this percentage consistently increased in HIV-infected individuals. While we have no obvious explanation for the discrepancy in CXCR5 expression on peripheral blood Vγ9Vδ2 T cells between these studies, in mice, CXCR5 expression during primary responses depends on sequential signaling by CD28 and OX40, suggesting the requirement for APCs [40], [41]. Hence, the presence or absence of DCs in the *in vitro* cultures might influence the outcome of CXCR5 expression. Thus, Vγ9Vδ2 T_FH_ cells differentiated *in vitro* with antigen and IL-21 can clearly express CXCR5, providing a molecular explanation for their clustering in germinal centres [20], [25]. Our present data also show that IL-21 plays a role in stimulating expression of the CXCR5 ligand, the chemokine CXCL13, by Vγ9Vδ2 T_FH_ cells. Overall, our results indicate that IL-21 drives Vγ9Vδ2 T cells to assume a T_FH_-like phenotype, thus evoking the crucial effect of IL-21 in the generation of CD4 T_FH_ cells [42]–[44]. Similar results have been published very recently by Bansal *at al.* [32], who have reported that Vγ9Vδ2 T cells stimulated with the phosphoantigen HMB-PP in the presence of IL-21, express markers associated with T_FH_ cells and support antibody production by B cells.

RETRACTED

Although these findings suggest that γδ T cells follow a similar differentiation pathway as conventional CD4 T_FH_ cells in their IL-21 requirement, expression of other important T_FH_ cell markers including PD-1, SAP, BTLA and CD57 is necessary to precisely define the Vγ9Vδ2 T_FH_ cell population. The determination of the co-expression of these markers is also important as this would resolve the proportion of the T_FH_ cell subset within the total Vγ9Vδ2 T cells derived from the *in vitro* culture. This is important for three reasons: (1) expression of two activations markers, CD25 and HLA-DR, rises the question of the heterogeneity of the *in vitro* activated Vγ9Vδ2 T cells; (2) it is not clear whether or not all Vγ9Vδ2 T cells can be biased towards a T_FH_ phenotype by IL-21, or are rather specific subsets of Vγ9Vδ2 T cells pre-programmed to become T_FH_-like cells and expand rapidly under the right conditions, as suggested by the heterogeneity of T_FH_-like Vγ9Vδ2 T cells in peripheral blood and tonsils [31]; (3) ICOS is not exclusively associated with T_FH_ functions [45]. In our experiments, only T_naive_ and a T_CM_ subsets of Vγ9Vδ2 T cells acquire some T_FH_ features when stimulated with IPP and IL-21 in the presence of irradiated DCs: since these subsets have the highest proliferative potential amongst Vγ9Vδ2 T cells [19], high ICOS expression after 12 days of culture should be the hallmark of their proliferation, rather than differentiation to a T_FH_ subset. Thus, differential ICOS expression by T_naive_/T_CM_ and/or T_FH_ subsets might also explain the observed trend with peak expression on day 4–6, and again on day 12.

IL-21 is the main cytokine shown to induce CD4 T_FH_ cells, but other cytokines have also been shown to induce T_FH_ cells, and these include IL-6, and IL-12. The requirements for the generation of conventional CD4 T_FH_ cells seem to be different for human and for mouse. While surprisingly in humans IL-12 also induces IL-21 production in a STAT-4-dependent manner [46], [47], in mouse IL-6 signaling also induces IL-21-secreting CD4 T_FH_ cells [44], [48]. Although we have not formally determined the signaling pathway that operates in Vγ9Vδ2 T_FH_ cells, data reported in Figure 2B clearly show that addition of IL-1β, IL-2, IL-6, IL-12, IL-15 or TGFβ, either alone, or in combination with IL-21, to cultures of Vγ9Vδ2 T cells and antigen did not induce or even enhance *BCL6* expression.

The acquisition of T_FH_-associated markers by Vγ9Vδ2 T cells and their dependence on IL-21 was initially suggested by microarray studies [25]. IL-21 turned out to have a similar capacity as the related cytokine IL-2 to support and sustain antigen-induced Vγ9Vδ2 T cell proliferation, yet without promoting the supposedly signatory cytokines IFN-γ and TNF-α [49], thus highlighting a much greater plasticity of Vγ9Vδ2 cell responses than previously appreciated [25]. While IL-21 may potentiate the cytolytic function of Vγ9Vδ2 T cells when combined with IL-2 [50], previous findings [25] and results here reported demonstrate that IL-21 on its own specifically co-stimulates expression of the chemokine receptor CXCR5, that enables T_FH_ cells to migrate into the B cell follicles, and also the CXCR5 ligand, CXCL13 that attracts further CXCR5^+^ cells, such as naive B cells and early activated CD4 T cells. As CXCR5 and CXCL13 are uniquely expressed in B cell follicles but mostly absent from extrafollicular areas, including the T zones of lymph nodes, spleen and Peyer’s patches, this implicates a role for IL-21-stimulated Vγ9Vδ2 T cells in orchestrating immune cell trafficking to the GCs.

RETRACTED

Differently than CD4 T_FH_ cells, Vγ9Vδ2 T_FH_ cells generated by culture with antigen and IL-21 do not produce IL-21, in agreement with previously published results [25]. On the other hand, the *in vitro* differentiated Vγ9Vδ2 T_FH_ cells have a Th2-type pattern of cytokine production upon short-term antigen stimulation *in vitro*, as they secrete IL-2, IL-4, and IL-10, but not IL-17, IFN-γ and TNF-α. This finding clearly contrasts with the cytokine production pattern of the Th1-like T_EM_ subsets of Vγ9Vδ2 T cells, which preferentially secrete IFN-γ and TNF-α [19]. The finding of a population of Vγ9Vδ2 T cells that secretes IL-4 and IL-10 is not new, and expands previous results demonstrating IL-4 production by resting [27], [51] and Vγ9Vδ2 clones [26], [52], most of which express CD27 (M. Bonneville and E. Scotet, unpublished observations). Moreover, and accordingly, we previously found that secretion of IL-4 and IL-10 was confined to the CD27^+^ subset of CXCR5^+^ Vγ9Vδ2 T cells [31]. However, Vγ9Vδ2 T_FH_ cells lack expression of GATA-3, and IL-13 mRNAs, both signatures of Th2 cells. The dissociated expression of IL-4 and IL-13/GATA-3 was unexpected but confirms a very recent paper in a mouse model of helminth infection [53], showing that IL-4, but not IL-13, was made by T_FH_ cells. In contrast, Th2 cells produced both cytokines. IL-13 production by Th2 cells was associated with large amounts of cellular transcription factor GATA-3, which was necessary for sustaining IL-13-producing. Conversely, T_FH_ cells produced only IL-4 and did not express GATA-3. Altogether, the results in mice and the data here reported in human Vγ9Vδ2 T_FH_ cells, indicate previously unappreciated regulation of these duplicated cytokines, as suggested by the differences between IL-4- and IL-13-expression in dependence on and expression of GATA-3.

It is likely that high levels of Bcl-6 expression in T_FH_ cells restrict GATA-3 to levels insufficient to activate *IL13*. Although Bcl-6 is a direct transcriptional repressor for many genes, it might suppress GATA-3 at a post-transcriptional level [37]. Because Bcl-6 overexpression can induce a T_FH_ phenotype [35], it is possible to speculate that decay of Bcl-6 or expression of Blimp-1 in T cells [36] is a prerequisite for relieving repression of the genetic programs, such as extended cytokine expression, necessary for the completion of Th2 differentiation in the periphery.

RETRACTED

Production of Th2-type cytokines together with expression of CD40L and ICOS strongly suggests that IL-21-stimulated Vγ9Vδ2 T cells are engaged in B cell activation and help for antibody production. Accordingly, we observed enhanced production of IgM, IgG and IgA when tonsillar B cells were coculturing with IL-21-stimulated Vγ9Vδ2 T_FH_ cells in the presence of Ag, thus fully identifying this cell population as a classical helper cells. Moreover, Ig production was consistently inhibited by blocking CD40-CD40L and ICOS-ICOSL interactions, or by neutralization of IL-4 or IL-10.

In theory one may argue that, due to the preactivation status of tonsillar B cells, Vγ9Vδ2 T_FH_ cells may only be active on already activated B cells and hence during secondary antibody responses. While we have no evidence to support or exclude such a possibility, our previous findings that circulating CXCR5^+^ Vγ9Vδ2 T cells are also able to help circulating naive B cells for antibody production [31], strongly suggests that Vγ9Vδ2 T_FH_ cells may play an important regulatory role in all aspects of humoral immunity.

γδ T cells have been reported to support antibody production in immunised and infected mice [11]–[14]. Of note, GCs are present in TCRαβ^−/−^ mice and develop in SCID mice upon adoptive transfer of γδ T cells and B cells, demonstrating that γδ T cells are sufficient to orchestrate follicular responses [11], [15], [54]. In humans, γδ T cells can be found in secondary lymphoid tissues [17], [18], where they are scattered throughout the T zone and clustered within GCs [18]–[20].

Contribution of Vγ9Vδ2 T_FH_ cells to antibody-mediated immune responses may occur early during microbial infections, before full development of acquired responses mediated by CD4 T cells. In humans, Vγ9Vδ2 T_CM_ cells are resident in the paracortical areas of lymph nodes, where they may become stimulated by antigen and express IL-21R: these, pre-activated cells may thus encounter IL-21 produced by CD4 T cells and as a consequence express a distinct set of molecules associated with providing B cell help. The interaction between with Vγ9Vδ2 T_FH_ cells, IL-21 producing CD4 T cells and B cells in reactive secondary lymphoid tissues is likely to impact on the production of high affinity antibodies against microbial pathogens.

In humans, the vast majority of Vγ9Vδ2 T cells directly recognize nonpeptide ligands without presentation by MHC molecules. Because αβ and γδ T cells recognize different types of antigens, the presence of a subset of each of these populations capable of inducing immunoglobulin secretion would provide a mechanism whereby humoral immune responses could be elicited against a diverse array of antigens irrespective of the type of responding T cell. Thus, the presence of Vγ9Vδ2 T cells in germinal centers would broaden the repertoire of antibodies produced by the B cell response.
